The article "Use of the Nuclear Matrix Protein 22 BladderChek Test for the Detection of Primary and Recurrent Urothelial Carcinoma" was published in 2020. Journal: Dis Markers.

# Use of the Nuclear Matrix Protein 22 BladderChek Test for the Detection of Primary and Recurrent Urothelial Carcinoma

**DOI:** 10.1155/2020/3424039

**Published:** 2020-05-08

**Authors:** Chang-sheng Xia, Chun-hong Fan, Ming Su, Qing-song Wang, Hui-zhang Bao

**Affiliations:** ^1^Department of Clinical Laboratory, Peking University People's Hospital, Beijing, China; ^2^College of Life Sciences, Peking University, Beijing, China

## Abstract

**Objective:**

To evaluate the performance of the nuclear matrix protein 22 (NMP22) BladderChek test in urothelial carcinoma (UC).

**Methods:**

We retrospectively analyzed 1318 patients who performed the NMP22 BladderChek tests. Of them, 103 were primary UC patients, 90 were surgical treatment UC patients, and 1125 were benign disease patients. The performance of the NMP22 BladderChek test for the diagnosis of primary and recurrent UC was evaluated. Moreover, the performance of urine cytology and the NMP22 BladderChek test for the diagnosis of primary UC was compared in 90 available subjects including 48 primary UC patients and 42 benign disease patients.

**Results:**

The sensitivity and specificity of the NMP22 BladderChek test were 37.9% and 95.8%, respectively, for the diagnosis of primary UC (*n* = 1228). The corresponding parameters of the NMP22 BladderChek test were 31.0% and 88.5%, respectively, for the diagnosis of recurrent UC (*n* = 90). The sensitivity and specificity of urine cytology were 54.2% and 97.6%, respectively, for the diagnosis of primary UC (*n* = 90); the corresponding parameters of the NMP22 BladderChek test were 41.7% and 83.3%, respectively; the corresponding parameters of the two tests combination were 64.6% and 83.3%, respectively. There was a significant difference in the performance between the NMP22 BladderChek test and urine cytology or the combination of two tests (*P* = 0.017 and 0.001, respectively).

**Conclusions:**

The NMP22 BladderChek test has a low sensitivity for detecting primary and recurrent UC. Urine cytology is superior to the NMP22 BladderChek test, and combined use of the two tests improves the sensitivity in the detection of primary UC.

## 1. Introduction

Urothelial carcinoma (UC) arises from the urothelium of the lower urinary tract (urethra and bladder) or the upper urinary tract (ureter and pyelocaliceal cavities). According to the National Cancer Institute of the United States, UC accounts for the vast majority (>90%) of bladder cancers. The estimated new cases and deaths from bladder cancer were 79030 and 16870 in the United States in 2017 [1]. Compared with the United States, the numbers were 80500 and 32900 in China in 2015 [2]. The current standard method for the detection of bladder cancer is an invasive cystoscopy. Urine cytology, the most accurate noninvasive test, is a secondary method after cystoscopy. Six urine tests for bladder cancer detection (UroVysion™, Immunocyt™, BTA stat, BTA TRAK, NMP22 ELISA, and NMP22 BladderChek) have received the US FDA approval [3], although none has sufficient accuracy to displace urine cytology [4]. Among these urine tests, only the NMP22 BladderChek test is approved by the Chinese FDA. The NMP22 BladderChek test is based on the detection of NMP22, a nuclear mitotic apparatus protein that is released from dead cells (e.g., apoptosis cells). In UC cells, NMP22 is elevated concordant with the structural and morphological change characteristic of malignant cell nuclei. So, the NMP22 BladderChek test can be used for the detection of UC. The NMP22 BladderChek test has been used in the clinic in China for several years. However, evaluation of the performance of this test is lacking. In the present study, we aimed to evaluate the performance of the NMP22 BladderChek test for the diagnosis of primary UC and compare its performance with urine cytology. In addition, the performance of the NMP22 BladderChek test for the detection of recurrent UC would be evaluated.

The article "Use of the Nuclear Matrix Protein 22 BladderChek Test for the Detection of Primary and Recurrent Urothelial Carcinoma" was published in 2020. Journal: Dis Markers.

## 2. Materials and Methods

### 2.1. Patients

We retrospectively reviewed all patients who performed the NMP22 BladderChek tests in the Department of Clinical Laboratory, Peking University People's Hospital from January 2015 to January 2017. Based on medical records, a total of 1318 patients were selected for this study. Of them, 103 were patients with primary UC, 90 were UC patients after surgical treatment, and 1125 were patients with benign diseases. Forty-eight primary UC patients and 42 benign disease patients performed urine cytology tests. For 90 UC patients with operational therapy, 9 patients performed urine cytology tests and 29 patients had recurrent UC. Among the benign disease patients, 40 had calculi, 485 hematuria, 231 urinary tract infection, 274 benign prostate diseases, 73 benign kidney diseases, and 22 benign bladder diseases. Patients were diagnosed as primary or recurrent UC based on cystoscopy and/or histopathological examination of biopsy and tumor tissue conducted in the Department of Pathology Laboratory at Peking University People's Hospital. UC stage was classified according to the TNM criteria, and grade was classified using the 2004 WHO/International Society of Urological Pathology (ISUP) consensus classification. The study was approved by the Institutional Review Board of Peking University People's Hospital.

### 2.2. Laboratory Analysis

The voided urine samples were collected from patients. The NMP22 BladderChek tests (Alere Scarborough, Inc., Maine, USA) were performed in the Department of Clinical Laboratory at Peking University People's Hospital, which was certified by the College of American Pathologists in 2015. The samples were tested and interpreted according to the manufacturer's instructions. Urine cytology performed in the Department of Pathology at Peking University People's Hospital was reported according to Paris classification. Cytology samples classified as positive in this study included those that were suspicious high-grade UC, low-grade UC, high-grade UC, and other type of cancer.

The article "Use of the Nuclear Matrix Protein 22 BladderChek Test for the Detection of Primary and Recurrent Urothelial Carcinoma" was published in 2020. Journal: Dis Markers.

### 2.3. Statistics

The continuous variable age was expressed as median (25^th^–75^th^ percentile). The Mann-Whitney *U* test was used to compare numerical data between two groups. Categorical variables were analyzed with a *χ*^2^ or Fisher's exact test and were shown as percentages. The McNemar test was performed to compare the diagnostic values among the NMP22 BladderChek test, urine cytology, and the combination of two tests. A *P* value of <0.05 was considered statistically significant. All statistical analyses were performed using SPSS software version 20.0. (SPSS, Inc., Chicago, IL).

## 3. Results

### 3.1. Patient Demographics and Clinical Characteristics

The patient demographics are shown in Table 1. Simply, the major patients with primary or recurrent UC were older men. The distributions of primary and recurrent UC according to site, stage, and grade are shown in Table 2. UC mainly occurred in the bladder, mainly in high-grade, and its stages mainly were Ta, T1, and T2.

### 3.2. Diagnostic Performance of the Urine Tests for the Diagnosis of Primary UC

Table 3 shows the diagnostic performance of the NMP22 BladderChek test, urine cytology, and the combination of two tests for the diagnosis of primary UC.

### 3.3. The Sensitivity of Urine Tests for the Diagnosis of Primary UC Stratified by Tumor Site, Invasivity, and Grade

Table 4 shows the sensitivity of the NMP22 BladderChek test and urine cytology for the diagnosis of primary UC stratified by tumor site, invasivity, and grade.

### 3.4. Comparison of Diagnostic Performance among the NMP22 BladderChek Test, Urine Cytology, and the Combination of Two Tests

Table 5 shows the comparison of diagnostic performance for the detection of primary UC among the NMP22 BladderChek test, urine cytology, and the combination of two tests based on clinical diagnosis.

### 3.5. Diagnostic Performance of the NMP22 BladderChek Test for the Detection of Recurrent UC

Table 6 shows the diagnostic performance of the NMP22 BladderChek test for the detection of recurrent UC.

### 3.6. The False-Positive Rate of the NMP22 BladderChek Test

For benign disease patients, the false-positive rate of the NMP22 BladderChek test was 4.2% (47/1125). The false-positive rates of the NMP22 BladderChek test were 20.0, 2.1, 6.9, 1.5, 2.7, and 31.8%, for the patients with urinary calculi, hematuria, urinary tract infections, benign prostate diseases, benign kidney diseases, and benign bladder diseases, respectively (*P* < 0.001).

The article "Use of the Nuclear Matrix Protein 22 BladderChek Test for the Detection of Primary and Recurrent Urothelial Carcinoma" was published in 2020. Journal: Dis Markers.

## 4. Discussion

Previous studies have reported the performance of the NMP22 BladderChek test and compared its performance with other urine tests including urine cytology for the detection of bladder cancer or UC [5–18]. For the diagnosis of primary bladder cancer or UC, the overall sensitivity and specificity of the NMP22 BladderChek test were from 16.7% to 70.5% and 40% to 100%, respectively. The corresponding data for the urine cytology was from 15.8% to 58.8% and 78% to 100%, respectively. For the detection of recurrent bladder cancer or UC, the overall sensitivity and specificity of the NMP22 BladderChek test were from 11% to 85% and 69.6% to 100%, respectively. There were significant differences in the performance of these two urine tests in these studies. The reasons for those discrepancies may be due to different study populations and different study designs.

In the present study, the sensitivity and specificity of the NMP22 BladderChek test for the diagnosis of primary UC in 1228 patients were 37.9% and 95.8%, respectively; the corresponding data in 90 patients were 41.7% and 83.3%, respectively. The difference in the specificity for two study populations may be due to benign disease patient selection bias. For urine cytology, the sensitivity and specificity for the diagnosis of primary UC in 90 patients were 54.2% and 97.6%, respectively. The combination of urine cytology and the NMP22 BladderChek test can increase the sensitivity to 64.6% while decreasing the specificity to 83.3%. For the detection of recurrent UC in 90 patients with surgical treatment, the sensitivity and specificity of the NMP22 BladderChek test were 31.0% and 88.5%, respectively. The sensitivities of the NMP22 BladderChek test and urine cytology for the detection of primary UC in our study were similar to those of O'Sullivan et al.'s study (37.9% and 56.1%, respectively) [14]. Our study shows that the sensitivities of the NMP22 BladderChek test and urine cytology for the diagnosis of primary UC are low and new more sensitive biomarkers should be used in the detection of UC. It is reported that Cxbladder has excellent sensitivity in the detection of primary and recurrent UC [14, 17].

Several studies have reported that the sensitivity of the NMP22 BladderChek test and urine cytology for the detection of UC increased when the stage or the grade rose [10, 18]. In our study, the sensitivity of the NMP22 BladderChek test and urine cytology for different tumor site, invasivity, and grade was analyzed. Firstly, we found that the sensitivity of the NMP22 BladderChek test in kidney UC was higher than that in bladder UC or ureter UC (69.2% vs. 30.9% or 26.7%). So, the NMP22 BladderChek test may be more applicable to use for detecting kidney UC. The sensitivity of urine cytology has no significant difference among kidney UC, ureter UC, and bladder UC. Secondly, our study showed that the sensitivity of the NMP22 BladderChek test increased as tumor invasivity or grade rose. The sensitivity of urine cytology increased as tumor grade rather than tumor invasivity rose.

The article "Use of the Nuclear Matrix Protein 22 BladderChek Test for the Detection of Primary and Recurrent Urothelial Carcinoma" was published in 2020. Journal: Dis Markers.

Previous studies have compared the performance of the NMP22 BladderChek test and urine cytology [5–18]. Our study showed the performance of urine cytology was superior to the NMP22 BladderChek test and the combination of two tests cannot improve the performance for detecting primary UC compared to urine cytology. However, the combination of two tests can increase the sensitivity in the diagnosis of primary UC.

Studies have reported that many factors can lead to false-positive results for the NMP22 BladderChek test [19, 20]. These factors included leukocytes, current use of blood pressure control drugs, urinary calculi, creatinine, recurrent urinary tract infections, and hematuria. In the present study, we found that benign bladder diseases and urinary calculi were the two most important factors for the false-positive results of the NMP22 BladderChek test. So, it is important to consider the influencing factors for interpreting the positive result of the NMP22 BladderChek test.

This study mainly evaluates the performance of the NMP22 BladderChek test for the diagnosis of primary UC with a large sample size. However, it has several limitations. First, it is a single-center and retrospective study. Second, not all patients performed urine cytology test. In the future, we will focus on resolving these issues by conducting a prospective multicenter study.

## 5. Conclusions

In conclusion, our study demonstrates that the NMP22 BladderChek test has a low sensitivity for the detection of primary and recurrent UC. Urine cytology is superior to the NMP22 BladderChek test, and the combination of two tests improves the sensitivity in the detection of primary UC. Moreover, new more sensitive biomarkers should be used in UC.

## Figures and Tables

**Table 1:** Patient demographics.

Group	Median age Year (25^th^–75^th^ percentile)	Male Number (%)
*n* = 1128^∗^		
Primary UC (*n* = 103)	66 (59-75)	70 (68.0%)
Benign diseases (*n* = 1125)	62 (52-72)	680 (60.4%)
*P* value	<0.001^†^	0.134^‡^
*n* = 90^#^		
Primary UC (*n* = 48)	69 (59-77)	33 (68.8%)
Benign diseases (*n* = 42)	59 (46-71)	24 (57.1%)
*P* value	0.002^†^	0.254^‡^
*n* = 90^&^		
Recurrent UC (*n* = 29)	75 (62-79)	21 (72.4%)
Nonrecurrent UC (*n* = 61)	64 (60-73)	38 (62.3%)
*P* value	0.010^†^	0.345^‡^

Note: UC, urothelial carcinoma; ^∗^patients performed the NMP22 BladderChek tests; ^#^patients performed the NMP22 BladderChek tests and urine cytology tests; ^&^patients with surgical treatment UC; ^†^the Mann-Whitney test was used to calculate two-sided *P* values; ^‡^categorical variables were analyzed with a *χ*^2^ test.

The article "Use of the Nuclear Matrix Protein 22 BladderChek Test for the Detection of Primary and Recurrent Urothelial Carcinoma" was published in 2020. Journal: Dis Markers.

**Table 2:** Distributions of primary and recurrent urothelial carcinoma by site, stage, and grade.

Site/stage/grade	Primary *n* = 103^∗^ Number (%)	Primary *n* = 48^#^ Number (%)	Recurrent *n* = 29 Number (%)
Site			
Bladder	68 (66.0%)	22 (45.8%)	29 (100.0%)
Ureter	15 (14.6%)	11 (22.9%)	0 (0.0%)
Renal pelvis	12 (11.6%)	9 (18.8%)	0 (0.0%)
Renal collecting duct	1 (1.0%)	1 (2.1%)	0 (0.0%)
Bladder and renal pelvis	2 (1.9%)	1 (2.1%)	0 (0.0%)
Bladder, ureter, and renal pelvis	1 (1.0%)	0 (0.0%)	0 (0.0%)
Ureter and renal pelvis	4 (3.9%)	4 (8.3%)	0 (0.0%)
Stage			
Ta	34 (33.0%)	8 (16.7%)	7 (24.1%)
T1	31 (30.1%)	15 (31.2%)	12 (41.4%)
T2	28 (27.2%)	20 (41.7%)	6 (20.7%)
T3+T4	10 (9.7%)	5 (10.4%)	4 (13.8%)
Grade			
PNLMP	9 (8.7%)	0 (0.0%)	0 (0.0%)
Low	29 (28.2%)	11 (22.9%)	5 (17.2%)
High	65 (63.1%)	37 (77.1%)	24 (82.8%)

Note: ^∗^patients performed the NMP22 BladderChek tests; ^#^patients performed the NMP22 BladderChek tests and urine cytology tests; PNLMP: papillary neoplasm of low malignant potential.

**Table 3:** Diagnostic performance of the urine test for the diagnosis of primary urothelial carcinoma.

Biomarker	Primary UC		%sensitivity (95% CI)	%specificity (95% CI)	%accuracy (95% CI)	%PPV (95% CI)	%NPV (95% CI)
	No. of patients						
	Yes	No					
*n* = 1228^∗^							
NMP22			37.9	95.8	91.0	45.3	94.4
Positive	39	47	(28.5-48.0)	(94.5-96.9)	(89.4-92.6)	(34.6-56.5)	(92.9-95.7)
Negative	64	1078					
*n* = 90^#^							
NMP22			41.7	83.3	61.1	74.1	55.6
Positive	20	7	(27.6-56.8)	(68.6-93.0)	(50.8-71.4)	(56.4-91.7)	(42.9-68.2)
Negative	28	35					
Cytology			54.2	97.6	74.4	96.3	65.1
Positive	26	1	(39.2-68.6)	(87.4-99.9)	(65.3-83.6)	(80.6-99.9)	(52.0-76.7)
Negative	22	41					
Combination			64.6	83.3	73.3	81.6	67.3
Positive	31	7	(49.5-77.8)	(68.6-93.0)	(64.0-82.6)	(65.4-92.4)	(52.7-79.8)
Negative	17	35					

Note: ^∗^patients performed the NMP22 BladderChek tests; ^#^patients performed the NMP22 BladderChek tests and urine cytology tests; UC, urothelial carcinoma; CI, confidence interval; PPV, positive predictive value; NPV, negative predictive value.

The article "Use of the Nuclear Matrix Protein 22 BladderChek Test for the Detection of Primary and Recurrent Urothelial Carcinoma" was published in 2020. Journal: Dis Markers.

**Table 4:** The sensitivity of urine tests for the diagnosis of primary urothelial carcinoma stratified by tumor site, invasivity, and grade.

	NMP22 positive Number (%)	Cytology positive Number (%)	*P* value^∗^
*n* = 103^∗^			
Site			0.010^†^; 0.772^‡^; 0.013^∮^; 0.024^§^
Bladder	21 (30.9%)		
Ureter	4 (26.7%)		
Kidney	9 (69.2%)		
Multisites	5 (71.4%)		
Invasivity			0.005
Nonmuscle invasive	18 (27.7%)		
Muscle invasive	21 (55.3%)		
Grade			0.001^&^; 0.006^※^
PNLMP	0 (0.0%)		
Low	6 (20.7%)		
High	33 (50.8%)		
*n* = 48^#^			
Site			0.635
Bladder		13 (59.1%)	
Ureter		4 (36.4%)	
Kidney		6 (60.0%)	
Multisites		3 (60.0%)	
Invasivity			0.790
Nonmuscle invasive		12 (52.2%)	
Muscle invasive		14 (56.0%)	
Grade			0.041
Low		3 (27.3%)	
High		23 (62.2%)	

Note: ^∗^patients performed the NMP22 BladderChek tests; ^#^patients performed the NMP22 BladderChek tests and urine cytology tests; PNLMP, papillary neoplasm of low malignant potential; ^∗^categorical variables were analyzed with a *χ*^2^ or Fisher's exact test; ^†^the sensitivity of the NMP22 BladderChek test was compared among bladder UC, ureter UC, kidney UC, and multisites UC; ^‡^bladder UC vs. ureter UC; ^∮^bladder UC vs. kidney UC; ^§^ureter UC vs. kidney UC; ^&^the sensitivity of the NMP22 BladderChek test was compared among PNLMP UC, low-grade UC, and high-grade UC; ^※^low-grade UC vs. high-grade UC.

**Table 5:** Comparison of diagnostic performance among the NMP22 BladderChek test, urine cytology, and the combination of two tests for the diagnosis of primary urothelial carcinoma based on clinical diagnosis.

Number of patients	Cytology		NMP22		*P* value
	Agreement	Disagreement	Agreement	Disagreement	
NMP22					0.017^∗^
Agreement	50	5			
Disagreement	17	18			
Combination					1.000^#^; 0.001^&^
Agreement	61	5	55	11	
Disagreement	6	18	0	24	

Note: the McNemar test was performed to compare the diagnostic values among the NMP22 BladderChek test, urine cytology, and the combination of two tests; ^∗^NMP22 vs. cytology; ^#^combination vs. cytology; ^&^combination vs. NMP22.

**Table 6:** Diagnostic performance of the NMP22 BladderChek test for the detection of recurrent urothelial carcinoma.

Biomarker	Recurrent UC		%sensitivity (95% CI)	%specificity (95% CI)	%accuracy (95% CI)	%PPV (95% CI)	%NPV (95% CI)
	No. of patients						
	Yes	No					
NMP22			31.0	88.5	70.0	56.2	73.0
Positive	9	7	(15.3-50.8)	(77.8-95.3)	(60.3-79.7)	(29.9-80.2)	(61.4-82.6)
Negative	20	54					

Note: UC, urothelial carcinoma; CI, confidence interval.

## Data Availability

The datasets used and/or analyzed during the current study are available from the corresponding author on reasonable request.
